The article "Zika Virus Prediction Using AI-Driven Technology and Hybrid Optimization Algorithm in Healthcare" was published in 2022. Journal: J Healthc Eng.

# Zika Virus Prediction Using AI-Driven Technology and Hybrid Optimization Algorithm in Healthcare

**DOI:** 10.1155/2022/2793850

**Published:** 2022-01-12

**Authors:** Pankaj Dadheech, Abolfazl Mehbodniya, Shivam Tiwari, Sarvesh Kumar, Pooja Singh, Sweta Gupta, Henry kwame Atiglah

**Affiliations:** ^1^Department of Computer Science and Engineering, Swami Keshvanand Institute of Technology, Management & Gramothan (SKIT), Jagatpura, Jaipur, Rajasthan-302017, India; ^2^Department of Electronics and Communication Engineering, Kuwait College of Science and Technology (KCST), Kuwait; ^3^Department of Computer Science and Engineering, Integral University, Lucknow, India; ^4^Department of Computer Science and Engineering, Babu Banarasi Das University, Lucknow, India; ^5^Department of Computer Science and Engineering, Amity School of Engineering and Technology, Noida, Sector-125, Uttar Pradesh, India; ^6^Department of CSE, School of Engineering and Technology, JLU, Bhopal, M.P, India; ^7^Department of Electrical and Electronics Engineering, Tamale Technical University, Tamale, Ghana

## Abstract

The Zika virus presents an extraordinary public health hazard after spreading from Brazil to the Americas. In the absence of credible forecasts of the outbreak's geographic scope and infection frequency, international public health agencies were unable to plan and allocate surveillance resources efficiently. An RNA test will be done on the subjects if they are found to be infected with Zika virus. By training the specified characteristics, the suggested Hybrid Optimization Algorithm such as multilayer perceptron with probabilistic optimization strategy gives forth a greater accuracy rate. The MATLAB program incorporates numerous machine learning algorithms and artificial intelligence methodologies. It reduces forecast time while retaining excellent accuracy. The projected classes are encrypted and sent to patients. The Advanced Encryption Standard (AES) and TRIPLE Data Encryption Standard (TEDS) are combined to make this possible (DES). The experimental outcomes improve the accuracy of patient results communication. Cryptosystem processing acquires minimal timing of 0.15 s with 91.25 percent accuracy.

## 1. Introduction

An infection's prelude and rapid spread to other regions of the globe attract the attention of the international community. Climate change is also a significant contributor to the rapid spread of illness. The species *Aedes aegypti*, which is widespread in urban areas, is the primary source of the illness, according to the CDC. Zika virus is a mosquito-borne illness that is comparable to dengue fever, west Nile virus, Chikungunya virus, and yellow fever, all of which are spread by mosquitoes. It is believed that mosquito bites are causing the spread of these illnesses and that *Aedes* mosquitoes are the primary vectors of these infections. Humans have had a significant challenge as a result of those, and this has mostly resulted in the transience of many tropical and subtropical nations [1]. It is an intrauterine illness caused by the Zika virus; the symptoms of Zika virus are often moderate fever, joint discomfort, and rashes, which are similar to those of dengue and Chikungunya virus. If an infected mosquito bites a pregnant woman and she becomes sick, the virus may spread across the placenta and affect the fetus. It is believed that pregnant women who are infected with the Zika virus will have neurological problems such as microcephaly and may give birth prematurely to their children. Even males who are infected with the 20 viruses may spread the virus to their sexual partners via anal, oral, or vaginal intercourse. The increasing population in urban areas has also increased the demand for water portability, which has resulted in people storing water in their homes, causing the *Aedes aegypti* mosquitoes to breed quickly in that climatic condition [2]. The increasing population in urban areas has also increased the demand for water portability, which has resulted in people storing water in their homes. It is believed that mosquitoes that have formed in water that we use in the home are the primary cause of the ailments. In India, the climatic conditions are ideal for mosquito breeding and development.

The article "Zika Virus Prediction Using AI-Driven Technology and Hybrid Optimization Algorithm in Healthcare" was published in 2022. Journal: J Healthc Eng.

Preventive methods for limiting the breading of mosquitoes in the infected region are part of the overall awareness campaign in the affected area: keeping the home clean, making sure there is no standing water in or around the house, and making sure any storage water is properly sealed with a lid if there is any. If any of them are discovered to be infected and exhibiting any of the symptoms, they must notify the appropriate healthcare facilities promptly. The individuals in question will be supplied with the medicine they need.

Cryptography is a critical milestone in the development of network security. The term cryptography refers to anything that is concealed or secret. Cryptography is the aim of secret writing with the goal of safeguarding information. The science of breaching cryptosystems, also known as cryptanalysis and cryptology, is the technique of breaking them down by trial and error. Cryptology plays a significant role in the protection of data in computer networks. Writing and solving data using codes are what cryptology is all about, and it includes both cryptography and cryptanalysis.

The article "Zika Virus Prediction Using AI-Driven Technology and Hybrid Optimization Algorithm in Healthcare" was published in 2022. Journal: J Healthc Eng.

Cryptography may be divided into three types: asymmetric, symmetric, and hashing. The following sections provide explanations of cryptography [3]. Asymmetric key cryptography is a kind of cryptography in which the key is not shared between two parties. Asymmetric cryptography, often known as public key cryptography, is distinguished by the fact that it uses both a public and a private key. While encrypting the data, the sender sends both the public key and the secret key used to decrypt the data. Only the person who has the secret key may decode the data throughout the decryption process. As a result, it is extremely safe when compared to the symmetric type, yet the time is extremely sluggish.  Figure 1 demonstrates the encryption process.

Having control over the data is regarded to constitute secure at the location where it is kept. If a user wants to make use of the advantages of cloud computing, he or she must first choose an appropriate network and then make use of the dispersed resources and arrangements made possible by cloud computing. When it comes to data transfer, the protection of the information is critical [4]. As a result, data that is really necessary should be secured, and obtaining privacy access rights is a major difficulty.  Figure 2 represents the data security issue.

### 1.1. Secureness in Cloud Database

Generally speaking, confidentiality refers to data or information that is not made available to anybody other than its owner, whether that is a person, a device, or a method. CSP is aware of the location or position of data stored by the user and knows where it is stored. There will be certain data that will provide some access assurance to a restricted number of people where the permission has been applied to particular data to secure data confidentiality in this case. Because of the sensitivity of the data that has been gathered in the cloud, some illegal access might result in risks. Assuredness should be provided to customers in the form of a privacy policy to ensure that data is handled appropriately and that mechanisms are in place to guarantee data security in the cloud. It is the responsibility of CSP to implement a variety of measures to ensure data integrity. The CSP informs the client about the kind of data that is being stored in the cloud [5]. As a result, it is necessary for CSP to maintain records about the data, such as the type of data, whether public or private, when and where it is required, the type of Virtual Memory and accumulated, the period of time when it is accessed, and so on, in order to protect the data from unauthorized access and to maintain data confidentiality.

### 1.2. Data Allocation in Server

We can access our data from any place and at any time thanks to the cloud, which is a superior service provider in our opinion. A risk is related with the location of data collection, which is associated with a higher degree of risk [6] as compared to other sites. The user should be aware of the location of sensitive data storage while an organization is using it, and he or she should have the ability to seek information about the location. At order to avoid confusion, the CSP and client should be in a certain place where the server location and data storage location are both known to the one in control of the scenario. When moving data from one location to another, such as via emails or uploaded photographs to Facebook, there are a number of things to take into account.

The article "Zika Virus Prediction Using AI-Driven Technology and Hybrid Optimization Algorithm in Healthcare" was published in 2022. Journal: J Healthc Eng.

### 1.3. Recovery of Input Data

While transferring data to the cloud, the CSP offers flexibility and ensures that the storage system has accurate information about the data sent. At the very least, a RAID configuration should be maintained in the storage system. The majority of CSPs will have several copies spread among a large number of independent or free servers. The cloud service provider provides the back-end application service, and in the event that a problem happens inside the company, the cloud service provider retrieves the data.

### 1.4. Secureness in Data Using Encryption Standards

According to a study report from 2100 Indian Business Technology Professionals, data auditing and confidentiality are the most significant obstacles in organizations using cloud technology [7]. The results of a survey conducted by Salt March Intelligence reveal the amount of sensitivity of business professionals to various technologies, including the difficulties they have in embracing cloud apps, infrastructures, customers, and storage. In today's fast-paced company climate, agility, cost savings, and flexibility are all required. The cloud environment provides all of these benefits. Zika virus illness prediction and data security are critical for both protecting patients from sickness and safeguarding their personal information. Nowadays, everything is being moved to the cloud, and healthcare is one of the industries that is being moved to the cloud. As a result, more precision in prediction is required; yet, only a limited amount of study has been done in order to anticipate the ZIKA virus. The amount of time it takes to perform a security request may vary depending on the configuration of the system or program being utilized. It is necessary to design a gap prediction and security algorithm in order to triumph over the research and to meet the requirements. In order to improve performance in forecasting the Zika virus with high levels of accuracy, the primary goal of the study activity is to develop new methods of prediction. Because there is no more data available, synthetic data is being generated for the prediction of the Zika virus. The data is divided into two groups based on the results of the machine learning classifier: infected and uninfected. For the prediction of the Zika virus, a variety of classifiers are tried; eventually, the MLP classifier outperforms the others in terms of accuracy. The use of encryption methods such as symmetric and asymmetric cryptography is investigated for the purpose of data security. For the purpose of encrypting the data, many methods are used. Finally, the suggested Hybrid Encryption technique is used for the purpose of safeguarding the data in the shortest amount of time possible, resulting in improved performance. The paper has the following structure: Section 2 consists of literature survey, Section 3 consists of methodology and outcome of proposed algorithm, and Section 5 consists of conclusions with future work.

The article "Zika Virus Prediction Using AI-Driven Technology and Hybrid Optimization Algorithm in Healthcare" was published in 2022. Journal: J Healthc Eng.

## 2. Literature Survey

Data integrity is discussed in detail by Wang et al. (2015) [8], who propose that when a service provider provides many services to cloud users and those users share data in a group, the originality of the data should be maintained, and this is accomplished through public auditing, in which case the signature of the shared data blocks must match the signature of the service provider. Different blocks are signed by different users at multiple times when different users modify the same file. For security reasons, any user may have their access terminated before they have the opportunity to be resigned by an existing user. It is necessary to invoke the idea of public auditing in conjunction with an efficient user revocation procedure; proxy resigns are carried out by the cloud on behalf of the current user at the moment of revocation. Existing users will not be required to download and resign their licenses. Chen et al. (2012) [9] have claimed that cloud computing offers several benefits, such as the ability to host applications and data on the client's behalf and that clients and users are increasingly using hybrid or public clouds. The scale of their market prevents certain huge organizations and corporations from shifting data to the cloud for some mission-critical applications, and this is a problem. Users' recommendations and perspectives on security and privacy protection concerns are taken into consideration, and appropriate measures are taken.

The authors provide a comprehensive analysis of data security and protection in relation to privacy regulations across the whole life cycle of data that is discussed in more detail. Some of the existing solutions and research efforts connected to privacy and security concerns are presented, as well as some of the challenges that remain. Lopez-Barbosa et al. (2016) [10] made a proposal about the real-time utilization of Internet of Things devices, such as smart phones. Using sensor devices and cloud computing, Quwaider and Jararweh (2016) [11] have presented a method for increasing public health-related awareness in the community. It is necessary to utilize the map reduction idea in order to detect anomalies in the information supplied by the sensors in real time. Mamun and colleagues (2017) [12] detailed how a notion of delivering speech signals to a doctor using cloud technology may be implemented. The doctor then diagnoses the patient and keeps track of them with the use of mobile phones and the cloud, which is the suggested methodology's manner of operation. With the use of smart phone technology, Zhang et al. [2015] [13] suggested a method of monitoring and managing the epidemic. Based on their network contacts, the whole population is divided into several clusters, with outbreak methodologies being employed and deployed at the cluster level in this case. Sareen, Sood, and Gupta (2016) [14] made a proposal for intrusive technical enhancement in the Internet of Things, mobile computing, among other things. In parallel with enhancing the quality of service provided by technology, healthcare services are also being enhanced. Because of this virus, people have been affected in a variety of geographical locations. As a result, a wide range of neurological symptoms and infections were discovered and documented. As a result, care should be made to avoid contracting Zika since it is very contagious among pregnant women, babies, and adults alike. The existence of the Zika virus in India was established by Sumit Bhardwaj and colleagues (2017) [15]. On the basis of the samples, four of the Zika-infected patients were identified during the screening process. As a result, it may become a significant concern in the future. When compared to Chikungunya, Zika is expected to become a major concern in the near future.

The article "Zika Virus Prediction Using AI-Driven Technology and Hybrid Optimization Algorithm in Healthcare" was published in 2022. Journal: J Healthc Eng.

The Zika epidemic, as represented by Petersen et al (2016) [16], as well as the infection among pregnant women and newborns, was addressed. Children with microcephaly are at a higher risk of developing neurological problems. A number of syndromes associated with neurological disorders were explored. This procedure has a high degree of accuracy, and the backpropagation approach was employed to anticipate the most accurate outcome possible. Kadri et al (2016) [17] have recommended that the Zika virus be designated a worldwide public health emergency. As a result, nations with a low risk of contracting the Zika virus were supplied with information pictorial expertise. It is necessary to take preventative measures.

It was suggested by Orellana et al. (2010) [18] that Google Docs have a new transparent user layer, which is implemented in Firefox, that encodes the record before collecting it in the Google server, making it impossible to access a data without having the correct password. The user is given the opportunity to choose the algorithms that will be used to encode the information. Once an algorithm has been chosen, the data is converted into cypher text and stored on Google's servers. The results demonstrate that blowfish performs much better when the key size is decreased, and the speed is increased. According to Singh et al. (2012) [19], elliptical curve cryptography is a fantastic approach of encryption technology. In wireless communication, the security layer must be implemented as robustly as possible, and for this reason, the framework is created using the ECC technique, which encrypts data in a powerful manner. It facilitates communication by using a multiagent system. The ECC has been used for the communication of wireless apps as well as certain web-based applications.

Singh et al. (2016) [20] have suggested a hybrid framework that incorporates both symmetric and asymmetric methods. When ECC and Blowfish are used together, the security level is significantly increased. The crypto and the CSP agent are both accessible for the purpose of distributing the key to the user. Even though CSP is not aware of it, the crypto agent is encrypting the data on its behalf. Only the authorized individual will be able to decipher the information. User's private key is shared with CSP, and CSP's public key is shared with the user. As a result, not even the CSP was able to decode the data. CA is in charge of providing these services. Nathiya et al. (2019) [21] provided an explanation of the many network assaults that might occur when a packet is being sent. The intrusion detection approach is explained here and divided into four stages, with the goal of detecting attacks on cloud data storage as the data is being transferred. When an attack is introduced into the network, it is detected using false alarm methods, and the suggested algorithm HINDS is used to identify the attackers who have done so. When it comes to cloud storage security, Gampala et al. (2012) [22] introduced the ECC method as well as a digital signature mechanism for protecting information. With the use of the ECC technique, the security of the data is enhanced while the key size is reduced.

The article "Zika Virus Prediction Using AI-Driven Technology and Hybrid Optimization Algorithm in Healthcare" was published in 2022. Journal: J Healthc Eng.

Jana et al. [23], in this case, used the hybrid approach, in which the downloading and uploading of data are completed at both the sender and recipient ends of the transmission. If any data is lost, it is impossible for both parties to decode it, which increases the overall security of the system. The multilayer algorithm is secure on both the user's and the server's end. Mohamed et al. (2015) [24] advocated that a framework be developed and validated for cloud environments in order to ensure that they are safe on both the client and server sides. When encoding or decoding data for connection setup, the Diffie Hellman cryptography is utilized in conjunction with ECC cryptography, and the integrity of the data is confirmed using the MD5 algorithm when updating the data. The suggested solution is a mix of ECC and SHA in order to provide a better outcome in data security. From the publications mentioned above, we can conclude that ECC is an improved asymmetric approach with a smaller key size. For the purpose of ensuring data integrity and authorization, a variety of encryption techniques and approaches were used. A brief overview of cloud computing is provided in the next chapter, followed by a detailed discussion of data security challenges and solutions for safeguarding data stored in the cloud.

## 3. Proposed Zika Virus Prediction Using MLP Classifier

Listed below is a description of each of the four components of the proposed system. The data gathering, fog layer, cloud layer, and, finally, the process are all in constant contact with the individuals engaged in the provision of healthcare. A framework has been designed for the identification of the Zika virus as well as the fortification of data in order to combat the virus. Cloud computing is used in this instance, because it is critical in the fact that it is capable of handling massive volumes of data from sensors and portable devices that have been mixed up. In order to connect end users to large-scale cloud services for storing and processing data, as well as for offering application services, it is essential to have a secure connection.  Figure 3 depicts the whole architecture of the predicted model for predicting the Zika virus, which includes all of its components.

### 3.1. Input Data Generation

Synthetic data is information that has been manufactured artificially rather than via real-world data collection. In algorithmic testing, it is used to evaluate a dataset of operational data or a dataset from a production environment. Additionally, it may be used to the validation of mathematical codes and, to a greater extent, to the training of machine learning forms. It is used in the modelling of a scenario or the calculation of a theoretical value, among other things. It delivers an unexpected outcome and if the findings are found to be unsuitable, it gives the required cures or answers to the problem. The actual and confidential data for the basic test are replaced with synthetic data created by the test engine. It is occasionally necessary to produce synthetic data in order to safeguard the confidentiality of the concerned data. We are utilizing synthetic data to test all of the real-time events that occur. We were unable to get real-time data because we needed to protect the anonymity of the patients who had been afflicted with the Zika virus; therefore, we developed synthetic data. Our technique is an early prediction system, and we are able to forecast whether a patient is infected or not based just on the symptoms that they exhibit. Even with that, we were unable to get real-time information. It is similar to a real-time dataset in that we create the information of the patients, such as how many days he has been sick with fever and whether he is travelling to a high-risk location. The symptoms of the Zika virus are thoroughly examined in order to develop the suggested technique for conducting the tests. Because it is difficult to get patient information in India, we want to employ synthetic data, which will allow us to test all of the possible combinations based on our assumptions. In this case, the diagnosis of infection is made based on seven separate symptoms. The potential combinations of Zika virus symptoms samples are included in the following. Then, using synthetic data, the location of mosquito breeding sites and the location of mosquito dense sites are determined. As a result, the mapping is done randomly with respect to the area, symptoms, and the user. Therefore, it is simple to distinguish between infected and uninfected patients, as well as the preventative actions that should be implemented by government agencies and hospital personnel [25].

The article "Zika Virus Prediction Using AI-Driven Technology and Hybrid Optimization Algorithm in Healthcare" was published in 2022. Journal: J Healthc Eng.

### 3.2. Input Data Tuning Layer

The suggested model includes a data component that comprises the specifics of the user's health data, environmental data, and location data, among other things. It is possible to get information on environmental conditions such as humidity, carbon dioxide level, and meteorological conditions by using environmental data. Because it is the primary cause of mosquito reproduction, it should be stressed repeatedly. Knowing well that our climatic conditions are ideal for mosquito reproduction, there is no need to watch everything every second. It is instead highlighted that the general climatic situation is favorable. The next step is to collect user health information. To do so, each user must register with the system using the mobile application that is available. Each user was assigned ID, which was generated. The indications of the Zika virus are obtained from users on a regular basis and reported to the authorities. The symptoms are responded in a yes or no fashion, according to the yes or no pattern. Not only are the symptoms recorded, but also is the user's health-related information. These kinds of information are gathered with the assistance of the sensor that is made available to the user [26]. The acquired data is protected using some kind of encryption technology, which is done in order of priority. User input is required for the symptoms of the Zika virus to be collected over a period of time, and the data are submitted as a yes or no pattern. The data collected by the environmental sensor includes information on mosquito breeding and population density. The sensor collects data in real time and uses it to pinpoint the location of the breeding grounds. In addition, carbon dioxide levels are regularly measured and studied in order to determine the climatic state of a certain site. Every piece of information pertaining to the environment is gathered in this section and saved in the fog computing servers. The data in the location part are connected to the data in the preceding section in that it displays the ideal site where there is a probability of mosquito density, and education opportunities are in height when compared to the climatic conditions.  Table 1 represents the attributes of the input used in the proposed work.

Table 2 gives the prediction rate based on the symptoms, and Table 3 represents prediction rate based on the environmental criteria.

### 3.3. Input Fog Computing Layer

Fog computing is a distributed computing environment that is used to handle large amounts of data in real time. It works as a platform between the cloud service provider and the user, allowing for large-scale data storage in the cloud to be accomplished. It is necessary to employ fog computing in order to reduce processing and performance time [27]. When it gathers all of the sensor data and stores it in a fog server, only the data that has been determined as necessary is evaluated and sent to the cloud for further processing. The processing speed and time are shortened as a result [28]. Because of the fog, the latency range, bandwidth, and everything else has risen. So, it serves as an independent server for data processing and archiving purposes. In the proposed work, fog is tasked with the responsibility of gathering all sensitive information from the user and determining if the symptoms match those of the user. As a consequence, this sort of result is solely sent to the cloud. Fog is a first-level environment in which sensitive data acquired from the sensor must be kept in huge quantities due to the nature of the environment. As a result, there is a need to analyze the data and ensure that they correspond to the given one. This is followed by sending the data to the cloud, where the final data categorization and subsequent processing will take place.

The article "Zika Virus Prediction Using AI-Driven Technology and Hybrid Optimization Algorithm in Healthcare" was published in 2022. Journal: J Healthc Eng.

### 3.4. Data Security

The acquired data are safeguarded via the use of a secret sharing method, in which the data are divided into little pieces and prioritizing is given for the various tiers. The level of protection provided for a piece of data is determined by its sensitivity. The protection of user personal data, which should be kept safe from the hands of unauthorized individuals, is given the highest priority. In the second level, there is information about the environment, and the information is saved on multiple servers. The third item is the least important since it should include information on symptoms as well as a warning to the individual to take the required precautions to prevent contracting the Zika virus. The hospitals in the government-run healthcare system provide the essential guidance to the public.  Figure 4 represents the overall proposed system.

### 3.5. Classification Using Multilayer Perceptron with Probability Optimization

The probabilistic model-based classifier is based on the mean and variance measures of the produced classes, which are a total of 124 classes in this case (62 classes of the NN and 62 classes of DT). The mean and variance measurements are used to calculate the exterior probability value of the approved picture, which is then expressed as a percentage. In order to avoid overfitting, we estimate the exterior probability of the 73 classes that are important to both the NN and the DT classifiers independently. The resulting probability of the NN classifier is multiplied by the resultant probability of the DT classifier to generate the new probability value for the classifier. The most exact recognition of the character picture is obtained in line with the greatest value of the new posterior probability distribution. The procedures involved in the modelling of the probabilistic classifier for the recognition of character are explored in further detail in the following sections.

In the probability calculation using (1),

(1) $$\begin{array}{c} \left(G\times 2\right)=\left[\begin{array}{cc} D_{0} & E_{f} \end{array}\right];\;1\leq o\leq 62. \end{array}$$

In this case, *o* is the output class label, and the class label of the NN classifier is indicated as Do, whereas the class label of the DT classifier is written as E. It is possible to define the mean and variance metrics associated with the NN and DT classifiers in the form of equations (2) and (3):

(2) $$\begin{array}{c} \text{Mean value }=o\times 2\left[\begin{array}{cc} N\left(D_{o}\right) & N\left(E_{o}\right) \end{array}\right], \end{array}$$

(3) $$\begin{array}{c} \text{Variance value }=o\times 2\left[\begin{array}{cc} W\left(D_{o}\right) & W\left(E_{o}\right) \end{array}\right]. \end{array}$$

The mean value is denoted by the letter N0, and the variance value is denoted by the letter W 0 in this equation. The 124 mean values are represented as o2, where 62 mean values correspond to the mean value of the NN classifier and the remaining 62 mean values correspond to the mean value of the DT classifier. Furthermore, the variance values of the NN and DT classifiers are computed and compared.

The article "Zika Virus Prediction Using AI-Driven Technology and Hybrid Optimization Algorithm in Healthcare" was published in 2022. Journal: J Healthc Eng.

NN classifier and DT classifier posterior probability formulas are shown in the following table: NN classifier posterior probability formula.

According to the following equation, the posterior probability formula for the NN classifier may be found:

(4) $$\begin{array}{c} Q\left(\frac{J}{D_{b}}\right)=\left[\frac{f\left[-\left({\left(D_{\text{b}}-N\left(D_{\text{B}}\right)\right)}^{2}/{\left(2+W\left(D_{\text{b}}\right)\right)}^{2}\right)\right]}{\sqrt{2*\pi *\;W\left(D_{\text{b}}\right)}}\right]. \end{array}$$

NN class label mean value is represented as M (C s), and NN class label variance measure is represented as W (D s) in this example.

According to the following equation, the posterior probability formula for the DT classifier may be found:

(5) $$\begin{array}{c} Q\left(\frac{J}{E_{b}}\right)=\left[\frac{\left[-\left({\left(E_{\text{f}}-N\left(E_{\text{f}}\right)\right)}^{2}/{\left(2*\text{ W}\left(E_{\text{f}}\right)\right)}^{2}\right)\right]}{\sqrt{2*\pi *\text{ W}\left(E_{\text{g}}\right)}}\right]. \end{array}$$

The mean value of the DT class label is denoted by the letter N (E o), while the variance measure of the DT class label is denoted by the letter W (E o).

NN classifiers have posterior probabilities that are higher than the posterior probability of the DT classifiers, which is represented by the formula for maximum posterior probability (max posterior probability) (5). The probabilistic model, as shown in equation (6), is used to identify the input character picture with the highest likelihood of being recognized:

(6) $$\begin{array}{c} D=\max_{b=1}^{62}\left|Q\left(I\;D\right)\right|. \end{array}$$

On the basis of the greatest measure of posterior probability, the identification of a character is conducted. In line with the acceptance criteria, the optical character picture with the highest likelihood of being identified properly is selected from the class.

The article "Zika Virus Prediction Using AI-Driven Technology and Hybrid Optimization Algorithm in Healthcare" was published in 2022. Journal: J Healthc Eng.

Figure 5 represents the Multilayer Perceptron Neural Network. Each of the NN and DT classifiers has its own mean value and variance value, which are computed independently in the algorithm. The posterior probability value is then computed using the method given above, which takes into account the mean and variance values that have been acquired. The posterior probability values of the NN and DT classifiers are merged to generate a single probability value, which is then blended with the other posterior probability values. Final recognition is achieved by using the greatest probability measure to determine whether or not the input character is recognized.

For identifying the instances, the multilayer perceptron classifier employs the backpropagation approach, which is described in more detail below. The network was built via the MLP algorithm, which was then analyzed and tweaked throughout the training phase. Except for the numeric classes, the network is composed entirely of sigmoid nodes for the threshold value. The backpropagation technique is required for the elements in order to get a complicated output result. It operates on the inputs in the network using the feedforward mechanism. When performing the iterative method, a set of weights is used to forecast the class label for each iteration. The feedforward algorithm contains a single input layer, one or more hidden layers, and eventually a single output layer, as shown in the diagram. During the classification process, if a mistake happens, the backpropagation approach is used to enhance the accuracy of classification while simultaneously decreasing the amount of input values and the time required for training.

(7) $$\begin{array}{c} {\text{layer}}_{l}=\;\sum y_{kl}z_{l}+\theta_{2},\\ P_{k}=y_{l}-\frac{1}{1+e^{-Ofl_{k}}}. \end{array}$$

It is computed by feeding the production spinal into the hidden film, which then processes the contribution over using the feedforwarding method, which results in a sigmoid function.

### 3.6. Weight and Objective Function of Classifier

The output node *k* has an activation value of and an anticipated target value of tk for node *k*, and the change among the predictable and authentic target values is represented as

(8) $$\begin{array}{c} B_{4}-B2-0, \end{array}$$

and node *k* is defined as

(9) $$\begin{array}{c} P_{2}={\overset{ˆ}{P}}_{2}Q_{2}\left(M-P_{2}\right),\\ \begin{array}{c} \Delta w_{jk}=4,\delta_{L}x_{6},\\ w_{jL}=w_{ja}+\Delta w_{jw}. \end{array} \end{array}$$

The network is recognized based on the pace at which it is learning. If it is set too low, network learning will be very sluggish, and if it is set too high, the network will oscillate between minimum and maximum values. Altering the knowledge rate from a big to a minor value during the backpropagation technique has a number of benefits. Assume that a network begins with weights that are far from the set of optimal weights and that it receives rapid training initially. When the learning rate falls throughout the course of learning, it is claimed that the process has reached a minimal optimum point. Because overshooting is less likely when the learning processes slow down.  Figure 6 shows the hybrid structure of AES with DES.

The article "Zika Virus Prediction Using AI-Driven Technology and Hybrid Optimization Algorithm in Healthcare" was published in 2022. Journal: J Healthc Eng.

The suggested hybrid technique includes two levels of encryption, or two tiers of security, and it is a framework that supports both symmetric encryption and asymmetric encryption functions at the same time. The two algorithms ECC and AES are a mix of hybrid methods for safeguarding data that are stored in the Common Security Policy (CSP). It is necessary to employ the AES symmetric method at the first level of encryption since the key is known to the user. The output of the first level of encryption is then encrypted a second time using the ECC algorithm, which is an asymmetric technique of encrypting data. In this case, the AES key is shared with both the user and the CSP in the first level, whereas in END USER Cloud Database Encryption using AES Level1 Encryption/Decryption using ECC Level 2 Data Collection the second level, the public key is used by the CSP and the private key is generated and shared with the user alone in the third level of the encryption scheme. The research of hybrid encryption method with two levels of encryption technology that went awry is shown in the illustration below. Each user will be provided with a set of two keys.

(10) $$\begin{array}{c} \text{Key }z=\text{AESj},\\ \text{Triple DES }Q_{J}\text{.} \end{array}$$

In this case, AESi represents the ith user of the symmetric key, and it is only known to the user. ECCpri displays the ith user's asymmetric private key, which is solely used by that particular user and no one else. The asymmetric public key user I is represented by the ECCpui, and it is known to the CSP. When a user saves data in the cloud, the cloud service provider (CSP) provides a set of keys that are used to encrypt the data. First, the data is encrypted using a key that is only known to the user and no one else. Before it is stored in the cloud storage, the cypher text generated as a consequence of the calculation is encrypted once again. In the next step, the completed encrypted text is saved in cloud storage [20–22]. Even the CSP is unaware of the key required to decode the data. In this case, the user will only be responsible for the first level of decryption. The key for second-level decryption is known to the user in this case. This process of delivering service to both the user and the CSP is carried out with the assistance of a third-party agent known as the Crypto Provider.

The article "Zika Virus Prediction Using AI-Driven Technology and Hybrid Optimization Algorithm in Healthcare" was published in 2022. Journal: J Healthc Eng.

Provider of cryptographic services: client-side encryption and decryption are handled by the client-side cryptographic processor (CP) [29]. It is ready after the set of users' keys has been collected. Whenever a CSP registers a new user, the CP makes the ECCpui available to the CSP. If a user wishes to keep data in cloud storage, he or she must first encrypt the data using the AESi algorithm and then using the ECCpui algorithm.

Pseudocode of Proposed work.

  Preparation of the references no and S (i);
  If (Refno = *n*), then the record already exists; else, the record does not exist.
  Alternately, update the user's information.
  Create a new entry in the database and save it there;
  If refno (updated data = old data) is true, then the values should be stored in the existing data.
  Else
  Keep track of the categorization value in the database;
  Change the patient's classification.
  In cases where S *i* corresponds to a *i*, where *i* ≥ *n* (number of patients), class C is equal to IN; otherwise, class C is equal to UIN.
  Inform the patient's infection classification;
  An alert has been sent to the doctor, the patient, and the hospitals.
  If the condition is met, the if statement is terminated.

## 4. Experimental Results

In order to make predictions about the Zika virus, the Matlab version is employed. It is a data mining software package that comprises a variety of machine learning algorithms for processing large amounts of data. It analyzes data in the ARFF file format by default, with CSV as a supported file format for Weka as a second option [30]. The explorer option is utilized for both the training set data and the testing dataset. The synthetic data was constructed using all feasible combinations of our assumptions and assumptions from other sources. Because it is regarded to be an uncommon illness in India, it is difficult to gather information about it.

Figure 7 represents the encrypted data. The MATLAB tool makes use of the dataset that was supplied in the previous section. It is necessary to utilize all of the possible combinations of the symptoms. Then, there are approximately 500 instances and 15 characteristics added to the mix. The individual is classed as infected or uninfected based on the information they provide. In this case, the MLP classifier is utilized to categorize the instances into groups. The MLP classifier has a 97 percent accuracy rate, which is excellent.

The article "Zika Virus Prediction Using AI-Driven Technology and Hybrid Optimization Algorithm in Healthcare" was published in 2022. Journal: J Healthc Eng.

The occurrences are classed as infected or uninfected based on the true positive and false positive rates for each case. The dataset under this study is publicly available. The algorithm for determining the sensitivity and specificity of the cases is used to determine these characteristics.

(11) $$\begin{array}{c} \text{Sensitivity}=\frac{\text{True Positive}}{\left(\text{True Positive}+\text{False Negative}\right)}\text{,}\\ \text{Accuracy}=\frac{\left(\text{True Negative}+\text{True Positive}\right)}{\left(\text{Tue Negative}+\text{True Positive}+\text{False Negative}+\text{False Positive}\right)}\text{.} \end{array}$$

Figure 8 represents the decrypted data. The threshold value for each class probability ranges from one class to the next. As a result, a classifier that yields an MLP threshold is described. It is indicated on the *X*-axis that the example dimensions are supplied and on the *Y*-axis that the true positive rate is presented.

Figure 9 represents the classification accuracy. Let us say that the sensitivity, specificity, and accuracy of the aforementioned equations are determined. It is determined whether or not the diagnostic test is accurate based on these data. Following that, the specificity of the test indicates the usual diagnostic situation, which is a negative result.  Table 4 provides an overview of the comparative examination of several classification algorithms.

While accuracy is defined as the ability to accurately detect the genuine result of the whole population, it is concerned with the real severity of a test diagnostic condition. A tall compassion test is designed to capture all of the potential positive situations that might occur during a test. As a result, sensitivity is utilized in the screening of diseases. When compared to other mosquito-borne diseases, the symptoms are mild to moderate. There is an incubation period of around 5 days for the virus [32]. If the symptoms linger for more than 7days, the individual should consult for an early prediction approach that employs our suggested method. If they are confirmed to be contaminated, they must have an RNA test in which their RNA is thoroughly examined and analyzed.

## 5. Conclusion

To determine whether or not the user is infected, the suggested system is utilized to gather data from the user and, depending on the symptoms, diagnose the user using the MLPNN algorithm for improved accuracy. The common characteristics of environmental factors are ready to be used to create a risky environment that is susceptible to infection. Once infections in patients have been found, the information pertaining to those diseases must be safeguarded in cloud storage. In order to safeguard the data stored in cloud storage, a double layer encryption approach using a hybrid crypto algorithm is used. The data is encrypted using the ECC and AES encryption methods, and even the third-party supplier has little knowledge of the contents of the encrypted data. Our suggested approach makes use of categorization to provide better results with an accuracy of 98 percent, and it assists the government's primary healthcare department in controlling the number of mosquitoes that are reproducing extremely successfully in the area. We are able to provide a better solution for the Zika virus infection when the healthcare industry and the government work together to implement our technology. The increased accuracy achieved in this research will be adopted, which means that it will assist physicians in the accurate prediction of Zika virus and the reduction of microcephaly illness in newborns and fetuses, among other things. Even premature delivery was averted to some extent. Patients in India must be monitored, and if any of the symptoms listed above are observed in any of them, the prediction system will take care of the prediction, as well as data protection, which is extremely secure, and the healthcare sectors do not essential to be concerned about the information being kept in fog storage because of the HEA used in the proposed model, which stands for Health Equity Act. Using the prediction system for anything beneficial to human civilization is the long-term goal of the project. The RNA test is the second step in the Zika virus prediction process. It is intended to concentrate on prevention and preventing the spread of the Zika virus. When it comes to cloud computing, new technologies are being developed on a daily basis, and data breaches are also occurring, so we must be prepared to deal with both the ups and downs. Because of this, research should be conducted for the benefit of society as a whole.

The article "Zika Virus Prediction Using AI-Driven Technology and Hybrid Optimization Algorithm in Healthcare" was published in 2022. Journal: J Healthc Eng.

## Figures and Tables

**Figure 1:** Asymmetric key encryption.

**Figure 2:** Data security issues.

**Figure 3:** Proposed model of Secured Zika Virus Prediction.

**Figure 4:** Overall flow of Proposed work using MLP Classifier.

**Figure 5:** Multilayer perceptron neural network. (a) Neural Network. (b) Deep neural network.

**Figure 6:** Hybrid AES with triple DES.

**Figure 7:** Encrypted data.

**Figure 8:** Decrypted data.

**Figure 9:** Classification accuracy.

**Table 1:** Input attributes collected to predict disease.

S.NO	Input	Description
1	S.No	Serial number of input user
2	Reg ID	Registration id of the user
3	Gender	Gender of the user
4	Name	Name of the input user
5	Location	Primary address of the patient
6	Contact no.	Emergency contact number

**Table 2:** Prediction criteria based on symptoms.

S.NO	Input attributes	Inputs
1	High fever	*N*/*y*
2	Conjunctivitis	*N*/*Y*
3	More joint pain	*N*/*Y*
4	Allergic reaction	*N*/*y*
5	Inner muscular pain	*N*/*y*
6	Headache, vomiting	*N*/*Y*
7	Overall risk criteria	

**Table 3:** Prediction criteria based on environmental hazards.

Attributes	Narration
Dense areas mosquito available	Value obtained from GPS location
Input breeding area	Value obtained from dense breed area
Humidity	Stagnant temperature
Temperature	Normal
Carbon di oxide	Higher level humidity

**Table 4:** Input classification table.

Author	Methods	Accuracy	Sensitivity	Specificity
Koc et al. 2014 [27]	LR	65	68	69
Hagan et al.1996 [28]	NN	83	84	85
Saren Sanjay 2017 [31]	NBN	87	80	73
Proposed method	MLP	97.5	97.63	96.28

## Data Availability

The data that support the findings of this study are available from the corresponding author upon request.

## References

[1] Kamal S. M., El Sayed Khalifa K. (2006). Immune modulation by helminthic infections: worms and viral infections. *Parasite Immunology*.

[2] Kumar K., Sharma A. K., Sarkar M., Chauhan A., Sharma R. (2014). Surveillance of *Aedes aegypti* (L.) mosquitoes in Mumbai international seaport (India) to monitor potential global health risks. *Journal of Insects*.

[3] Diffie W., Hellman M. (1976). New directions in cryptography. *IEEE Transactions on Information Theory*.

[4] Alcaraz C., Zeadally S. (2013). Critical control system protection in the 21st century. *Computer*.

[5] El Ghazouani M., El Kiram M. A., Er-Rajy L. (2019). Blockchain & multi-agent system: a new promising approach for cloud data integrity auditing with deduplication. *International Journal of Communication Networks and Information Security*.

[6] Garbarino E., Strahilevitz M. (2004). Gender differences in the perceived risk of buying online and the effects of receiving a site recommendation. *Journal of Business Research*.

[7] Ryoo J., Rizvi S., Aiken W., Kissell J. (2013). Cloud security auditing: challenges and emerging approaches. *IEEE Security & Privacy*.

[8] Wang Q., Wang C., Ren K., Lou W., Li J. (2010). Enabling public auditability and data dynamics for storage security in cloud computing. *IEEE Transactions on Parallel and Distributed Systems*.

[9] Luo S., Lin Z., Chen X., Yang Z., Chen J. Virtualization security for cloud computing service.

[10] Lopez-Barbosa N., Gamarra J. D., Osma J. F. (2016). The future point-of-care detection of disease and its data capture and handling. *Analytical and Bioanalytical Chemistry*.

The article "Zika Virus Prediction Using AI-Driven Technology and Hybrid Optimization Algorithm in Healthcare" was published in 2022. Journal: J Healthc Eng.

[11] Quwaider M., Jararweh Y. (2015). Cloudlet-based efficient data collection in wireless body area networks. *Simulation Modelling Practice and Theory*.

[12] Sondhi S., Saad S., Shi K., Mamun M., Traore I. (2021). Chaos engineering for understanding consensus algorithms performance in permissioned blockchains. https://arxiv.org/abs/2108.08441.

[13] Yu N. H., Hao Z., Xu J. J., Zhang W. M., Zhang C. (2013). Review of cloud computing security. *Acta Electonica Sinica*.

[14] Sareen S., Gupta S. K., Sood S. K. (2017). An intelligent and secure system for predicting and preventing Zika virus outbreak using Fog computing. *Enterprise Information Systems*.

[15] Gupta P., Bharadwaj S., Sharma V. K. A survey to bridging the gap between energy and security in IoT and home.

[16] Petersen W. A., Rutledge S. A. (1998). On the relationship between cloud-to-ground lightning and convective rainfall. *Journal of Geophysical Research: Atmospheres*.

[17] Benarous L., Kadri B. (2021). Obfuscation-based location privacy-preserving scheme in cloud-enabled internet of vehicles. *Peer-to-Peer Networking and Applications*.

[18] Rodrıguez-Silva D. A., González-Castano F. J., Adkinson-Orellana L., Fernández-Cordeiro A., Troncoso-Pastoriza J. R., González-Martınez D. Encrypted Domain Processing for Cloud Privacy.

[19] Singh S., Jeong Y.-S., Park J. H. (2016). A survey on cloud computing security: Issues, threats, and solutions. *Journal of Network and Computer Applications*.

[20] Singh A., Juneja D., Malhotra M. (2015). Autonomous agent based load balancing algorithm in cloud computing. *Procedia Computer Science*.

[21] Nathiya T., Suseendran G. (2019). An effective hybrid intrusion detection system for use in security monitoring in the virtual network layer of cloud computing technology. *Data Management, Analytics and Innovation*.

[22] Gampala V., Inuganti S., Muppidi S. (2012). Data security in cloud computing with elliptic curve cryptography. *International Journal of Soft Computing and Engineering*.

[23] Jana B., Chakraborty M., Mandal T. (2019). A task scheduling technique based on particle swarm optimization algorithm in cloud environment. *Soft Computing: Theories and Applications*.

[24] Mohamed E. M., Abdelkader H. S., El-Etriby S. Enhanced data security model for cloud computing.

[25] Li X., Zheng Y., Alshehri M. D. (2021). Cognitive AmBC-noma IoV-MTS networks with IQI: reliability and security analysis. *IEEE Transactions on Intelligent Transportation Systems*.

[26] Anderson L. M., Scrimshaw S. C., Fullilove M. T., Fielding J. E., Normand J., Task Force on Community Preventive Services (2003). Culturally competent healthcare systems. *American Journal of Preventive Medicine*.

The article "Zika Virus Prediction Using AI-Driven Technology and Hybrid Optimization Algorithm in Healthcare" was published in 2022. Journal: J Healthc Eng.

[27] Samanta D., Karthikeyan M. P., Karuppiah D. (2021). Optimized tree strategy with principal component analysis using feature selection-based classification for newborn infant’s Jaundice symptoms. *Journal of Healthcare Engineering*.

[28] Rajawat A. S., Bedi P., Goyal S. B. (2021). Fog big data analysis for IoT sensor application using fusion deep learning. *Mathematical Problems in Engineering*.

[29] Dey B. L., Pandit A., Saren M., Bhowmick S., Woodruffe-Burton H. (2016). Co-creation of value at the bottom of the pyramid: analysing Bangladeshi farmers’ use of mobile telephony. *Journal of Retailing and Consumer Services*.

[30] Li∗ X., Zhao M., Zeng M. (2021). Hardware iab systems: reliability and security. *IEEE Transactions on Communications*.

[31] Koç M. L., Koç D. I. (2020). A cloud theory based reliability analysis method and its application to reliability problems of breakwaters. *Ocean Engineering*.

[32] Hagan M., Siddiqui F., Sezer S., Kang B., McLaughlin K. Enforcing policy-based security models for embedded SoCs within the internet of things.

